RETRACTED

# Linc00152 promotes malignant progression of glioma stem cells by regulating miR-103a-3p/FEZF1/CDC25A pathway

**DOI:** 10.1186/s12943-017-0677-9

**Published:** 2017-06-26

**Authors:** Mingjun Yu, Yixue Xue, Jian Zheng, Xiaobai Liu, Hai Yu, Libo Liu, Zhen Li, Yunhui Liu

**Affiliations:** 1 Department of Neurosurgery, Shengjing Hospital of China Medical University, Shenyang, 110004 People’s Republic of China; 2 Liaoning Clinical Medical Research Center in Nervous System Disease, Shenyang, 110004 People’s Republic of China; 3 Key Laboratory of Neuro-oncology in Liaoning Province, Shenyang, 110004 People’s Republic of China; 4 Department of Neurobiology, College of Basic Medicine, China Medical University, Shenyang, 110122 People’s Republic of China; 5 Key Laboratory of Cell Biology, Ministry of Public Health of China, China Medical University, Shenyang, 110122 People’s Republic of China; 6 Key Laboratory of Medical Cell Biology, Ministry of Education of China, China Medical University, Shenyang, 110122 People’s Republic of China

**Keywords:** Long non-coding RNA, linc00152, miR-103a-3p, Glioma stem cells, FEZF1, CDC25A

## Abstract

**Background:**

Glioma is one of the most frequent intracranial malignant tumors. LncRNAs have been identified as new modulators in the origination and progression of glioma.

**Methods:**

Quantitative real-time PCR were conducted to evaluate the expression of linc00152 and miRNA-103a-3p in glioma tissues and cells. Western blot were used to determine the expression of FEZF1 and CDC25A in glioma tissues and cells. Stable knockdown of linc00152 or over-expression of miR-103a-3p in glioma stem cells (GSCs) were established to explore the function of linc00152 and miR-103a-3p in GSCs. Further, luciferase reports were used to investigate the correlation between linc00152 and miR-103a-3p. Cell Counting Kit-8, transwell assays, and flow cytometry were used to investigate the function of linc00152 and miR-103a-3p in GSC malignant biological behaviors. ChIP assays were employed to ascertain the correlations between FEZF1 and CDC25A.

**Results:**

Linc00152 was up-regulated in glioma tissues as well as in GSCs. Knockdown of linc00152 inhibited cell proliferation, migration and invasion, while promoted GSC apoptosis. Linc00152 regulated the malignant behavior of GSCs by binding to miR-103a-3p, which functions as a tumor suppressor. In addition, knockdown of linc00152 down-regulated forebrain embryonic zinc finger protein 1 (FEZF1), a direct target of miR-103a-3p which played an oncogenic role in GSCs. FEZF1 elevated promoter activities and up-regulated expression of the oncogenic gene cell division cycle 25A (CDC25A). CDC25A over-expression activated the PI3K/AKT pathways, which regulated the malignant behavior of GSCs.

RETRACTED

**Conclusions:**

Linc00152/miR-103a-3p/FEZF1/CDC25A axis plays a novel role in regulating the malignant behavior of GSCs, which may be a new potential therapeutic strategy for glioma therapy.

**Electronic supplementary material:**

The online version of this article (doi:10.1186/s12943-017-0677-9) contains supplementary material, which is available to authorized users.

## Background

Glioma is one of the most frequent intracranial malignant tumors. Due to the highly invasive growth pattern and frequent resistance to therapies, the prognosis for patients with glioma is dismal [1]. Glioma stem cells (GSCs), a neoplastic subpopulation within glioma, are responsible for therapy resistance [2] and poor survival rate of glioma [3]. GSCs have characteristics of neurosphere formation, self-renewal and multi-directional differentiation [4]. Therefore, illustration of the molecular mechanisms underlying GSCs offers new orientation toward the gloma treatments.

Lately, long non-coding RNAs (lncRNAs), which are defined as non-coding RNAs more than 200 nucleotides in length, are involved in various genetic phenomena, including transcriptional, post-transcriptional and epi-genetic regulations [5]. Moreover, lncRNAs have been identified as new modulators in the origination and progression of glioma [6]. Mounting evidence has also demonstrated that lncRNAs involved in the regulation of gene expression in stem cell biology and in tumorigenesis [7].

Long intergenic non-coding RNA 152 (Linc00152) was found aberrant expression in numerous cancers. Linc00152 was distinctly up-regulated in gastric cancer and its expression was positively correlated with tumor invasion depth, lymph node metastasis and poor survival [8]. Moreover, linc00152 could modulate the expression of miR-193a-3p to increase disease recurrence through acting as a competing endogenous RNA in colon cancer [9]. However, the expression and possible functional role of linc00152 in GSCs remains uncharted.

MicroRNAs (miRNAs) are small non-coding RNAs that regulate gene expression by binding to the 3′-UTRs of mRNAs [10]. MiRNAs are reported to be involved in a variety of human carcinogenesis, including glioma [11]. MiR-103a-3p was illuminated to participate in the proliferation, migration and invasion process in ovarian carcinoma [12]. It is predicted that miR-103a-3p has putative binding sites with linc00152 by Starbase (http://starbase.sysu.edu.cn/). Moreover, miR-103a-3p was identified as prognostic biomarker of colon cancer, breast cancer and pleural mesothelioma [13–15], etc. However, limited knowledge is available concerning whether miR-103a-3p affected the biological processes of GSCs.

RETRACTED

Forebrain embryonic zinc finger protein 1(FEZF1) is highly conserved transcription factor that encoded a transcriptional repressor which contributed to the embryonic migration of gonadotropin-releasing hormone neurons into the brain [16]. In addition, FEZF1 is required for olfactory development and knock down FEZF1 in mice, olfactory neurons fail to mature [17]. We predicted FEZF1 as a presumed target of miR-103a-3p by miRNA target prediction software Target Scan (http://www.targetscan.org/). Studies have shown that FEZF1 played a oncogenic role through DNA demethylation [18] in gastric cancer. Nevertheless, the role of FEZF1 in GSCs remains ambiguous.

Cell division cycle 25A (CDC25A), a member of the CDC25 family of phosphatases, removes the inhibitory phosphorylation in cyclin-dependent kinases (CDKs) [19], and regulates the progression from G1 to the S phase of the cell cycle [20]. It is discovered that the promoter of CDC25A contains sequence of CnnCAnCn core which is a putative consensus FEZF1 binding site [21, 22]. Furthermore, CDC25A was identified as an oncogene, and over-expression of CDC25A promoted tumorigenesis [23].

The major purpose of this study was to explore the expression of linc00152, miR-103a-3p, FEZF1 and CDC25A in glioma tissues and GSCs. We also investigated the roles in regulating the malignant behavior of GSCs and the potential molecular pathways among them. Our findings will give a new direction for the treatment of glioma.

## Results

### Isolation and identification of GSCs

As shown in Additional file 1: Figure S1A, GSCs-87 (or GSCs-251) isolated from glioma cells were cultured in the serum-free medium and formed cell spheres. Immunofluorescence analysis indicated that most cells within spheres were positive to neural stem cell lineage markers Nestin and CD133 (Additional file 1: Figure S1B). During the differentiation assay, single-cell suspensions of spheres were differentiated and stained with GFAP and β-tubulin III, implying that isolated GSCs-87 and GSCs-251 possessed the potential for differentiation toward astrocytic and neuronal lineages (Additional file 1: Figure S1C).

### Linc00152 expression was up-regulated in glioma tissues and GSCs while miR-103a-3p was down- regulated in glioma tissue and GSCs

The linc00152 and miR-103a-3p expression levels in normal brain tissues(NBTs), grade I-II (low grade) and grade III-IV (high grade) glioma tissues, as well as in GSCs and non stem cells (non-GSCs) were evaluated by qRT-PCR. As shown in Fig. 1a-b, linc00152 expression levels elevated with the pathological grades of glioma tissues and were apparently up-regulated in GSCs compared with non-GSCs. However, expression of miR-103a-3p was negatively correlated with the progression of glioma pathological grade and was distinctly down-regulated in GSCs compared with non-GSCs (Fig. 2a-b).

RETRACTED

**Fig. 1:** linc00152 functioned as an oncogene in GSCs. **a** Expression of linc00152 in glioma tissues of different grades and normal brain tissues (NBTs). (Data are presented as the mean ± SD (*n* = 10, each group). **P < 0.01 vs. NBTs group; *P < 0.05 vs. low grade group; ^*#*^ *P* < 0.05 vs. low grade group. **b** Expression of linc00152 in non-GSCs and GSCs (Data are presented as the mean ± SD (*n* = 5, each group). **P < 0.01 vs. non-GSCs-U87 group; ^*##*^ *P* < 0.01 vs. non-GSCs-U251 group. **c** Relative expression of linc00152 after GSCs transfected with sh-linc00152 plasmids and scrambled vectors (NC). **d** CCK-8 assay was conducted to explore the proliferation effect of linc00152 on GSCs. **e** Limiting dilution assay showing the impact of linc00152 on the sphere-formation ability of GSCs. **f** Transwell assays for assessing GSC migration and invasion. Typical images and accompanying statistical plots were presented. **g** Flow cytometry detected the apoptosis of GSCs with the knockdown of linc00152. Data are presented as the mean ± SD (*n* = 5, each group). *P < 0.05 vs. sh-NC group. Scale bars represent 20 μm. The photographs were taken at 200 × magnification

**Fig. 2:** miR-103a-3p manifested an anti-oncogene in GSCs. **a** Expression of miR-103a-3p in glioma tissues of different grades and NBTs (Data are presented as the mean ± SD (*n* = 10, each group). **P < 0.01 vs. NBTs group; *P < 0.05 vs. NBTs group; ^*#*^ *P* < 0.05 vs. low grade group. **b** Expression of miR-103a-3p in non-GSCs and GSCs (Data are presented as the mean ± SD (*n* = 5, each group). **P < 0.01 vs. non-GSCs-U87 group; ^##^ *P* < 0.01 vs. non-GSCs-U251 group. **c** Relative expression of miR-103a-3p after GSCs transfected with pre-miR-103a-3p, anti-miR-103a-3p as well as their scrambled vectors (NC). **d** Effect of miR-103a-3p on the proliferation of GSCs. **e** Effect of miR-103a-3p on the sphere-formation ability of GSCs. **f** Effect of miR-103a-3p on the migration and invasion of GSCs. **g** The apoptotic rates after GSCs transfected with pre-miR-103a-3p and anti-miR-103a-3p. *P < 0.05 vs. pre-NC group; ^*#*^ *P* < 0.05 vs. anti-NC group. Scale bars, 20 μm. The photographs were taken at 200 × magnification

### Knockdown of linc00152 repressed malignant biological properties of GSCs

Following the evaluation of linc00152 expression in GSCs, we further explored the possible effect of linc00152 on the proliferation, migration, invasion and apoptosis of GSCs. Stable linc00152 silenced constructs were used to appraise the function of linc00152 on GSCs. The RT-PCR assay was applied to demonstrate the linc00152 knockdown (Fig. 1c). The Cell Counting Kit-8 (CCK-8) assay suggested that GSCs proliferation was declined in the sh-linc00152 group than that in the sh-NC group (Fig. 1d). The limiting dilution assay implied that knockdown of linc00152 hindered the sphere-formation ability of GSCs (Fig. 1e). The migration and invasion of GSCs assay showed that the numbers of migrated and invaded cells in the sh-linc00152 group were significantly decreased compared with the sh-NC group (Fig. 1f). Flow cytometry analysis implied that silence of linc00152 markedly increased apoptosis of GSCs (Fig. 1g). Taken together, linc00152 functioned as an oncogene in GSCs.

RETRACTED

### miR-103a-3p manifested a tumor suppressor

Had appraised the miR-103a-3p expression in GSCs, we assessed the effect of miR-103a-3p on GSCs and transfected miR-103a-3p-agomir (pre-miR-103a-3p) and miR-103a-3p-antagomir (anti-miR-103a-3p) into GSCs, respectively. The RT-PCR assay was applied to detect the transfection efficiency of miR-103a-3p (Fig. 2c). As shown in Fig. 2d, pre-miR-103a-3p group emerged a significantly declined proliferation in GSCs compared to the pre-NC group. The limiting dilution assay implied that over-expression of miR-103a-3p hindered the sphere-formation ability of GSCs (Fig. 2e). Transwell assays implied that migrated and invaded cell numbers were remarkably decreased in pre-miR-103a-3p group than in pre-NC group (Fig. 2f). Flow cytometry analysis suggested that over-expression of miR-103a-3p markedly promoted apoptosis of GSCs (Fig. 2g). The results above inferred that miR-103a-3p, in contrast to linc00152, appeared as tumor-suppressive function in GSCs.

### Linc00152 is a direct target of miR-103a-3p

Increasing evidence implied that lncRNAs could be competing endogenous RNAs (ceRNAs) or molecular sponges in affecting the expression and biological functions of miRNAs [24]. Using a bioinformatics database (Starbase), linc00152 harbor one conjectural binding site of miR-103a-3p. To certify the prediction that miR-103a-3p could directly bind to linc00152, we detected the expression of miR-103a-3p in sh-linc00152 GSCs by qRT-PCR. MiR-103a-3p expression was raised in the sh-linc00152 group whereas not in the sh-NC group. In comparison, linc00152 expression declined in the pre-miR-103a-3p group comparing with the pre-NC group (Fig. 3a). In addition, the correlation between expression of linc00152 and miR-103a-3p in glioma tissues was detected by qRT-PCR. As shown in Fig. 3b, miR-103a-3p expression was negatively correlated with linc00152 expression. The best fit slope was −4.243 (*P* < 0.01). Dual-luciferase gene reporter assays were employed to assess the binding sites of linc00152 and miR-103a-3p. The luciferase activity was dramatic decline in the linc00152-wt + miR-103a-3p group than in the Control group (Fig. 3d), while there was no distinction between the linc00152-mut + miR-103a-3p group and the Control group in luciferase activity, indicating the presence of a binding site between linc00152 and miR-103a-3p. In summary, linc00152 is a direct target of miR-103a-3p and there might be a reciprocal repression feedback loop between linc00152 and miR-103a-3p.

RETRACTED

**Fig. 3:** Reciprocal restrain between miR-103a-3p and linc00152, down-regulated of linc00152 hindered the malignant behavior of GSCs by target miR-103a-3p. **a** qRT-PCR analysis revealed the negative correlation between miR-103a-3p and linc00152 expression in glioma cells. **P < 0.01 vs. pre-NC group; ^*##*^ *P* < 0.01 vs. anti-NC group; **P < 0.01 vs. sh-NC group. **b** Linear regression analysis was done to each individual linc00152 and miR-103a-3p expression, the slope was −4.243, **P < 0.01. **c** Schematic representation of the putative binding site for linc00152 and miR-103a-3p, and the contrivable mutant sequence indicated for the reporter assay. **d** The relative luciferase activities were restrained in the HEK-293 T cells co-transfected with vector linc00152-wt and miR-103a-3p. *P < 0.05. vs. linc00152-wt + miR-103a-3p-NC group; ^*#*^ *P* < 0.05. vs. linc00152-mut + miR-103a-3p-NC group. **e** The CCK-8 assay was conducted to evaluate the effects of linc00152 and miR-103a-3p on the proliferation of GSCs. **f**-**g** The capacities of migration and invasion were detected through transwell assays on GSCs. **h** Flow cytometry analysis of GSCs in groups according to linc00152 and miR-103a-3p expression. *P < 0.05 vs. sh-NC + pre-NC group; ^*#*^ *P* < 0.05 vs. sh-linc00152 + pre-NC groups;^*&*^ *P* < 0.05 vs. sh-NC + pre-miR-103a-3p group; ^▲^ *P* < 0.05 vs. sh-NC + anti-NC group; ^★^ *P* < 0.05 vs. sh-linc00152 + anti-NC group;^▼^ *P* < 0.05 vs. sh-NC + anti-miR-103a -3p group. Scale bars, 20 μm. For **a**, **c**, **d**, **e** and **g**, data are presented as the mean ± SD (*n* = 5, each group)

### MiR-103a-3p involved in the tumor-suppressive effects of linc00152 knockdown in GSCs

Ulteriorly, to explore the tumor-suppressive effects of linc00152 knockdown were mediated by miR-103a-3p, GSCs were divided into nine groups: the Control group, the sh-NC + pre-NC group (cells stably expressing sh-NC, co-transfected with pre-NC), sh-linc00152 + pre-NC group (cells stably expressing sh-linc00152, co-transfected with pre-NC), sh-NC + pre-miR-103a-3p group (cells stably expressing sh-NC, co-transfected with pre-miR-103a-3p), sh-linc00152 + pre-miR-103a-3p group (cells stably expressing sh-linc00152, co-transfected with pre-miR-103a-3p), sh-NC + anti-NC group (cells stably expressing sh-NC, co-transfected with anti-NC), sh-linc00152 + anti-NC group (cells stably expressing sh-linc00152, co-transfected with anti-NC), sh-NC + anti-miR-103a-3p group (cells stably expressing sh-NC, co-transfected with anti-miR-103a-3p) and sh-linc00152 + anti-miR-103a-3p group (cells stably expressing sh-linc00152, co-transfected with anti-miR-103a-3p). CCK8 assay indicated that GSCs proliferation was significantly decreased in the sh-linc00152 + pre-NC group, sh-NC + pre-miR-103a-3p group and sh-linc00152 + pre-miR-103a-3p group than the sh-NC + pre-NC group, respectively (Fig. 3e). Moreover, the numbers of GSC migration and invasion were dramatically declined in the sh-linc00152 + pre-NC group, sh-NC + pre-miR-103a-3p group and sh-linc00152 + pre-miR-103a-3p group than in the sh-NC + pre-NC group, respectively (Fig. 3f-g). In addition, GSCs of sh-linc00152 + pre-NC group, sh-NC + pre-miR-103a-3p group and sh-linc00152 + pre-miR-103a-3p group manifested higher apoptosis rates compared with the sh-NC + pre-NC group, respectively (Fig. 3h). The data above implied that miR-103a-3p mediated the tumor suppressive effects of linc00152 knockdown in GSCs.

RETRACTED

### FEZF1 was involved in the linc00152/miR-103a-3p dependent malignant progression of GSCs

The above results uncovered that linc00152 and miR-103a-3p have remarkable impacts on the biological behaviors of GSCs, but the latent molecular mechanisms remain blurry. Bioinformatics database (Targetscan) speculated that several genes would be downstream targets of miR-103a-3p, including FEZF1. Next, we appraised the impact of linc00152 or miR-103a-3p on mRNA and protein levels of FEZF1 by qRT-PCR and western blot, and noticed expression level of FEZF1 was prominently affected among the predicted downstream genes of miR-103a-3p. Then, the expression level of FEZF1 in GSCs was explored, which was transfected with sh-linc00152, pre-miR-103a-3p or anti-miR-103a-3p. As shown in Fig. 4a and c, expression of FEZF1 was declined in the sh-linc00152 group comparing with the sh-NC group. On the contrary, cells in anti-miR-103a-3p group manifested higher levels of FEZF1 than those in anti-NC group (Fig. 4b and d).

**Fig. 4:** FEZF1 was a target gene of miR-103a-3p, the expression of FEZF1 was regulated by both linc00152 and miR-103a-3p. **a** qRT-PCR analysis of the effect of linc00152 on FEZF1 mRNA expression in glioma cells. **P < 0.01 vs. sh-NC group. **b** qRT-PCR analysis of the effect of miR-103a-3p on FEZF1 mRNA expression in glioma cells. **P < 0.01 vs. pre-NC group; ^*##*^ *P* < 0.01 vs. anti-NC group. **c** Western blot analysis on FEZF1 in linc00152-knockdown GSCs, with GAPDH as an endogenous control. *P < 0.05 vs. sh-NC group. **d** Western blot analysis for expression between miR-103a-3p and FEZF1 in GSCs, with GAPDH as an endogenous control. *P < 0.05 vs. pre-NC group; ^*#*^ *P* < 0.05 vs. anti-NC group. **e** Western blot analysis for FEZF1 in GSCs co-transfected with sh-linc00152 and pre-miR-103a-3p or anti-miR-103a-3p, with GAPDH as an endogenous control. *P < 0.05 vs. sh-NC+ pre-NC group. ^*#*^ *P* < 0.05 vs. sh-linc00152 + pre-NC group; ^*&*^ *P* < 0.05 vs. sh-NC + pre-miR-103a-3p group; ^▲^ *P* < 0.05 vs. sh-NC + anti-NC group; ^★^ *P* < 0.05 vs. sh-linc00152 + anti-NC group; ^▼^ *P* < 0.05 vs. sh-NC + anti-miR-103a -3p group. For **a**-**e**, data are presented as the mean ± SD (*n* = 5, each group). **f** Schematic representation of the putative binding site for miR-103a-3p and FEZF1, and the contrivable mutant sequence for the reporter assay. **g** The relative luciferase activities were hindered in the HEK-293 T cells co-transfected with vector pre-miR-103a-3p and FEZF1-wt. *P < 0.05. vs. FEZF1-wt + pre-NC group

In addition, FEZF1 expression was lower in the sh-linc00152 + pre-NC group, sh-NC + pre-miR-103a-3p group and sh-linc00152 + pre-miR-103a-3p group comparing with the NC group, repectively (Fig. 4e). The data above indicated that FEZF1 was involved in the linc00152/miR-103a-3p dependent malignant progression of GSCs.

RETRACTED

### FEZF1 was up-regulated in glioma tissues and GSCs, and facilitated GSC proliferation, migration and invasion and receded GSC apoptosis

After verified FEZF1 was a target of miR-103a-3p, we investigated the protein levels of FEZF1 in NBTs, glioma tissues and GSCs by Western blot. As shown in Fig. 5a-b, FEZF1 protein levels elevated with the pathological grades of glioma tissues and were apparently up-regulated in GSCs compared with non-GSCs. In consequence, we conjectured that FEZF1 facilitated the malignant progression of GSCs and detected the effect of FEZF1 on the proliferation, migration, invasion and apoptosis of GSCs. As shown in Fig. 5c, the CCK8 assay implied that proliferation of GSCs was raised in the FEZF1(+) groups compared with the FEZF1(+)-NC group. Transwell assays indicated that migration and invasion capacity of GSCs in the FEZF1(+) group were stronger than that in the FEZF1(+)-NC group (Fig. 5d). Further, up-regulated FEZF1 dramatically suppressed apoptosis in GSCs compared with the NC group (Fig. 5e).

RETRACTED

**Fig. 5:** FEZF1 was up-regulated in glioma tissues, and played an oncogenic role in GSCs. **a** FEZF1 protein expression in non-tumorous brain tissues, low-grade glioma tissues (WHO I-II), and high-grade glioma tissues (WHO III-IV), with GAPDH as an endogenous control. Data are presented as the mean ± SD (*n* = 10, each group). **P or ^*##*^ *P <* 0.01 vs. non-tumorous brain tissue group. **b** Western blot analysis of FEZF1 expression in non-GSCs and GSCs, with GAPDH as an endogenous control. **P < 0.01 vs. non-GSC group. **c** CCK8 assay was performed to evaluate the effect of FEZF1 on the proliferation of GSCs. **d** Quantification of GSC migration and invasion upon FEZF1 over-expression or down-regulation. Representative images and accompanying statistical plots are presented. **e** Flow cytometry analysis of the effects of FEZF1 on GSCs. Data are presented as the mean ± SD (*n* = 5, each group). *P < 0.05 vs. FEZF1 (+)-NC group; ^*#*^ *P* < 0.05 vs. FEZF1(−)-NC group. Scale bars, 20 μm. The photographs were taken at 200 × magnification. **f** Effect of FEZF1 on the CDC25A protein expression, with GAPDH as an endogenous control. Data are presented as the mean ± SD (*n* = 5, each group). *P < 0.05 vs. FEZF1(+)-NC group, ^*#*^ *P* < 0.05 vs. FEZF1(+)-NC group. **g** Effect of FEZF1 on the CDC25A mRNA expression. Data are presented as the mean ± SD (*n* = 5, each group). *P < 0.05 vs. FEZF1(+)-NC group, ^*#*^ *P* < 0.05 vs. FEZF1(+)-NC group. **h** Schematic depiction of the CDC25A reporter constructs used and the luciferase activity. The Y-bar shows the position of the deletions on the DNA fragments. X-bar shows the constructed plasmid activity after normalization with the co-transfected reference vector (pRL-TK), and relative to the activity of pEX3 empty vector,which the activity was set to 1. Data representmeans ± SD (*n* = 5, each). **i** Schematic representation of the CDC25A promoter region 3000 bp upstream of the transcription start site (TSS) which designated as +1. ChIP PCR products for putative binding sites and an upstream region not expected to associate with FEZF1 are depicted with bold lines. Immunoprecipitated DNA was amplified by PCR. Normal rabbit IgG was used as a negative control

### miR-103a-3p hindered FEZF1-induced malignant behavior on GSCs by targeting its 3′-UTR

To further affirm whether FEZF1 is a direct target of miR-103a-3p, luciferase assay was carried out. Luciferase activity was dramatically declined in cells co-transfected with pre-miR-103a-3p and FEZF1-wt (Fig. 4g), illustrated that FEZF1 was a direct target of miR-103a-3p. Nevertheless, there was no significant difference between FEZF1-mut + pre-miR-103a-3p group and FEZF1-mut + miR-103a-3p-NC group, suggesting the specific binding site of miR-103a-3p in the FEZF1- 3′-UTR.

RETRACTED

Furthermore, to explore whether miR-103a-3p suppressed GSC malignant evolution were mediated by FEZF1, down-regulated FEZF1 by pre-miR-103a-3p was rescued using FEZF1 prior to the assessment of the cell proliferation, migration, invasion and apoptosis. CCK8 assay indicated that miR-103a-3p over-expression restrained the proliferation of GSCs, whereas FEZF1 over-expression accelerated the proliferation of GSCs. FEZF1 over-expression rescued the inhibitory effect of miR-103a-3p over-expression on the proliferation of GSCs (Fig. 6b). Besides, transwell assay revealed that miR-103a-3p over-expression impaired the migrating and invading capacity of GSCs, while FEZF1 over-expression showed the contrary result. FEZF1 over-expression rescued the impaired migration and invasion of GSCs induced by miR-103a-3p over-expression (Fig. 6c). Further, flow cytometry analysis implied that over-expression of miR-103a-3p promoted apoptosis of GSCs, whereas over-expression of FEZF1 suggested the opposite result. FEZF1 over-expression rescued the enhancement of miR-103a-3p over-expression on the apoptisis of GSCs (Fig. 6d). These results revealed that FEZF1 mediated the tumor-suppressive effects of miR-103a-3p over-expression on GSCs.

**Fig. 6:** miR-103a-3p inhibited malignant progression of GSCs by binding to the FEZF1 3′-UTR. **a** Effect of miR-103a-3p and FEZF1 co-transfection on the CDC25A mRNA expression. **b** The CCK-8 assay was used to assess the effects of miR-103a-3p and FEZF1 on GSC proliferation. **c** Transwell assay was employed to detect the effects of miR-103a-3p and FEZF1 on GSC migration and invasion. Representative images and accompanying statistical plots are presented. **d** Flow cytometry analysis of GSCs in groups according to miR-103a-3p and FEZF1(+) expression. **e** Effect of miR-103a-3p and FEZF1 co-transfection on the CDC25A, p-AKT and p-PI3K protein expression, with GAPDH as an endogenous control. *P < 0.05 vs. pre-NC + FEZF1 -NC group, ^*#*^ *P* < 0.05 vs. pre- miR-103a-3p + FEZF1-NC group. Scale bars, 20 μm. The photographs were taken at 200 × magnification. Data are presented as the mean ± SD (*n* = 5, each group)

### FEZF1 up-regulated the promoter activities and bound to the promoters of CDC25A in GSCs

The results above revealed that FEZF1 exerted oncogenic role by facilitating malignant biological behaviors of GSCs. However, the underlying molecular mechanism remains indistinct. Both FEZF1 and FEZF2 belong to the forebrain embryonic zinc finger (Fez) family [25], and as previous report, CnnCAnCn core, which was found in promoter region of CDC25A by DBTSS database (http://dbtss.hgc.jp/), was identified as putative consensus FEZF2 binding site [21]. In addition, FEZF1 and FEZF2 were reported to have the same target gene [22]. Therefore, we hypothesized FEZF1 could bind with CDC25A.

RETRACTED

Recent research identified CDC25A as an oncogene and over-expression of CDC25A promoted a variety of tumors. CDC25A was observed high expression in lung cancer [26, 27] and high expression of CDC25A predicted poor prognosis in human lung adenocarcinoma [28]. Moreover, up-regulation of CDC25A was reported to enhance cell proliferation, which possibly mediated chemoresistance in human AML [29]. To confirm whether CDC25A was regulated by FEZF1 in GSCs, qRT-PCR and western blot analysis was carried out.

As shown in Fig. 5f-g, expression of CDC25A protein and mRNA were enhanced in FEZF1(+) group comparing with FEZF1 (+)-NC group. In GSCs co-transfected with miR-103a-3p and FEZF1, miR-103a-3p over-expression declined mRNA and protein expression of CDC25A, whereas FEZF1 over-expression increased the expression (Fig. 6a and e).

To verify whether FEZF1 is necessary for the promoter activity of CDC25A in GSCs, a suite of constructs were generated and luciferase assays were applied. The promoter sequences of CDC25A were set according to the database of DBTSS HOME (http://dbtss.hgc.jp/). By analyzing these DNA sequences in the 3000 bp region upstream of the transcription start site (TSS) and its 100 bp downstream sequence, we confirmed two putative FEZF1 binding sites in CDC25A (Fig. 5i). So a suite of DNA fragments were constructed and ligated into the pGL3 basic vector. Wild-type, deletion construct and putative FEZF1 binding sites were indicated. After co-transfection with pEX3-FEZF1, deletion of the −707 site region significantly decreased the promoter activities of CDC25A. The results indicated that the responsive FEZF1-binding sites resided within −707 site region of CDC25A (Fig. 5h).

To explore whether FEZF1 directly associated with the promoters of CDC25A in GSCs, ChIP assay was applied. As a negative control, PCR was performed to amplify the 2000 bp upstream region of the putative FEZF1 binding site which was not supposed to associate with FEZF1. Our results showed that there was direct association of FEZF1 with putative binding site 2 of CDC25A. There was no association of FEZF1 with putative binding site 1 of CDC25A and the control regions (Fig. 5i). These results revealed that FEZF1 could up-regulate the promoter activities and bind to the promoter of CDC25A.

### CDC25A accelerated malignant biological behaviors of GSCs by promoting the PI3K/AKT pathway

Up-regulated of CDC25A was discovered in human glioma specimens and depletion of CDC25A suppressed cell proliferation and induced apoptosis in glioma cell lines [30]. The results above implied a tumor promotion of CDC25A in glioma. However, the effect of CDC25A in GSCs was fuzzy. Hence, we detected the protein level of CDC25A in GSCs. As shown in Fig. 7a, CDC25A protein levels elevated dramatically in GSCs compared with the non-GSCs. Furthermore, we evaluated the effect of CDC25A on the proliferation, migration, invasion and apoptosis of GSCs. As shown in Fig. 7b-c, over-expression of CDC25A promoted the proliferation, migration and invasion capacity of GSCs. Further, up-regulated CDC25A distinctly diminished apoptosis in GSCs compared with the NC group (Fig. 7d).

RETRACTED

**Fig. 7:** CDC25A was up-regulated in GSCs, and played an oncogenic role in GSCs. **a** Western blot analysis of CDC25A expression in non-GSCs and GSCs, with GAPDH as an endogenous control. *P < 0.05 vs. non-GSCs-U87 group, ^*#*^ *P* < 0.05 vs. non-GSCs-U251 group. **b** CCK8 assay was performed to evaluate the effect of CDC25A on the proliferation of GSCs. **c** Quantification of GSC migration and invasion upon CDC25A overexpression or downregulation. Representative images and accompanying statistical plots are presented. **d** Flow cytometry analysis of the effects of CDC25A on GSCs. **e** Western blot analysis of the PI3K/AKT pathway regulated by CDC25A in GSCs. Data are presented as the mean ± SD (*n* = 5, each group). *P < 0.05 vs. CDC25A (+)-NC group; ^*#*^ *P* < 0.05 vs. CDC25A (−)-NC group. Scale bars, 20 μm. The photographs were taken at 200 × magnification

The results above illustrated CDC25A promoted the proliferation, migration and invasion in GSCs, and refrained the apoptosis of GSCs. To investigate the underlying molecular mechanism, we assessed the activity of PI3K/AKT pathway by Western blot assays. As shown in Fig. 7e, over-expression of CDC25A prompted the p-PI3K and p-AKT expression in GSCs. Besides, in GSCs co-transfected with miR-103a-3p and FEZF1, miR-103a-3p over-expression declined expression of CDC25A, P-AKT and P-PI3K, whereas FEZF1 over-expression increased the expression (Fig. 6e). These results demonstrated that CDC25A accelerated malignant biological behaviors of GSCs by promoting the PI3K/AKT pathway.

### Linc00152 knockdown combined with over-expressed miR-103a-3p suppressed tumor growth and manifested high survival in nude mice

To further certify the above findings, an in vivo tumor model was employed. The results indicated that the linc00152 knockdown, miR-103a-3p over-expression, and linc00152 knockdown combined with over-expressed miR-103a-3p groups had smaller tumors compared with the linc00152(−)-NC + miR-103a-3p(+)-NC group (Fig. 8a-c). In addition, tumors in the linc00152(−) + miR-103a-3p(+) group manifested the smallest volume compared to the other groups (Fig. 8a-c). Moreover, mice in the linc00152(−) + miR-103a-3p(+) group had the longest survival time (Fig. 8d).

RETRACTED

**Fig. 8:** Tumor xenografts study of tumor growth and survival rates in nude mice. **a** The nude mice carrying tumors of respective groups were shown. **b** Sample tumors from respective group were shown. **c** Tumor growth curves of five groups in nude mice (*n* = 8). Tumor growth was monitored for up to 40 days. *P < 0.05 vs. linc00152(−)-NC + miR-103a-3p(+)-NC group, ^*#*^ *P* < 0.05 vs. linc00152(−) group, ^*▲*^ *P* < 0.05 vs. miR-103a-3p(+) group. **d** Survival curves of nude mice injected into the right striatum. Mice were monitored for up to 50 days (*n* = 8). **e** The schematic cartoon of the mechanism of linc00152 as an oncogene by regulating miR-103a-3p/FEZF1/CDC25A pathway in glioma stem cells

## Dicussion

In this study, we elaborated that expression of the lncRNA linc00152 was elevated in glioma tissues and GSCs. Linc00152 could directly bind to miR-103a-3p and negatively regulated the expression of miR-103a-3p. This implied a significant mechanism of linc00152 pathway in the glioma intervention. Knockdown of linc00152 restrained proliferation, migration and invasion, and facilitated apoptosis in GSCs. On the contrary, miR-103a-3p manifested carcinostatic role in GSCs and suppressed the proliferation, migration and invasion, prompted apoptosis of GSCs. In addition, FEZF1 was identified as a direct target of miR-103a-3p and mediated the tumor-suppressive effects of miR-103a-3p. Moreover, inhibition of miR-103a-3p promoted the expression of CDC25A by up-regulating FEZF1, which positively control the promoter activities via binding to the promoter of CDC25A. Further, PI3K/AKT pathway was blocked when CDC25A was suppressed. Experiment in vivo showed that knockdown of linc00152 combined with over-expression of miR-103a-3p generated the smallest tumor and led to the longest survival time in nude mice.

Glioblastoma (GBM) is one of the most common and lethal primary malignant brain tumor in adults [31, 32]. GBM harbor a subpopulation of self-renewing, therapy-resistant cells, GSCs, which can flourish in the stresses present in an unfavorable tumor microenvironment [33]. In consequence, therapies targeting GSCs have become a hotspot in treatment of glioma [34]. A growing number of evidence has implied that lncRNAs play an important role in the occurrence and progression of tumors recently. Exploring the potential molecular mechanisms of lncRNAs in GSCs may provide promising therapeutic strategies in glioma.

RETRACTED

Our present data revealed that linc00152 was positively correlated with the histopathological grade in human glioma tissues and elevated in GSCs. In addition, knockdown of linc00152 inhibited cell proliferation, migration and invasion, as well as promoted apoptosis in GSCs, which indicated that linc00152 may serve as an oncogene in GSCs. Previous researches also showed the same oncogenic function of linc00152. Cai Q reported linc00152 was up-regulated in gallbladder cancer and correlated negatively with the overall survival time in gallbladder cancer patients [35]. In addition, linc00152 was identified as increased expression in gastric cancer [36] and regarded as a novel biomarker for predicting gastric cancer [37]. Our results illustrated that linc00152 acted as a oncogene in GSCs for the first time, but the underlying mechanisms need to be investigated.

LncRNAs finely regulate gene expression through a variety of ways, including transcriptional regulation, splicing and translation, post-transcriptional regulation and epitogenetic modulation, etc. [38]. To detect the potential oncogenic mechanism of linc00152 in glioma, bioinformatics analysis software was applied to identify miR-103a-3p as a novel target of linc00152. MiR-103a-3p situated in 5q34, and was associate with tumor, Parkinson disease and pregnancy-related complications [39–41]. Our study suggested that miR-103a-3p was declined in glioma tissues and GSCs compared with NBTs and glioma cells, respectively. Furthermore, over-expression of miR-103a-3p inhibited proliferation, migration and invasion, as well as promoted apoptosis in GSCs. This was consistent with the previous studies showing that miR-103a-3p was low expressed in gastric cancer [42] as well as bladder carcinoma [43], and played a crucial role in cancer suppression.

Mechanistically, miR-103a-3p was identified as a direct target of linc00152 by dual-luciferase assay, suggesting the potential reciprocal repression feedback loop between linc00152 and miR-103a-3p. In addition, our results showed that ablation of linc00152 inhibited cell proliferation, migration and invasion as well as inducing apoptosis in GSCs by elevating miR-103a-3p, implying that linc00152 knockdown impaired the malignant behavior of GSCs by up-regulating miR-103a-3p. Moreover, the in vivo studies showed that nude mice in the sh-linc00152 + pre-miR-103a-3p group manifested the smallest tumors and highest survival compared to the other groups, suggesting that these were likely to achieve synergistic anti-tumor effects. Collectively, linc00152 acted as an oncogenic gene by restraining miR-103a-3p in GSCs, but the further mechanisms under miR-103a-3p were blurred.

RETRACTED

We discovered that the protein levels of FEZF1 had adverse changes to the alteration of miR-103a-3p. Luciferase reporter assays certified that miR-103a-3p regulated gene expression post-transcriptionally by binding to the 3’UTR of FEZF1. In addition, our research showed that FEZF1 expression was raised in glioma tissues as well as in GSCs. Over-expression of FEZF1 facilitated cell proliferation, migration and invasion, and inhibited cell apoptosis, implying that FEZF1 functions as an oncogene in GSCs. Consistent with our results, FEZF1 was reported over-expressed in gastric cancer tissues and played a significant role in the progression and metastasis of gastric cancer by activation of the K-ras oncogene [44]. What’s more, miR-103a-3p and FEZF1 co-overexpression significantly rescued the inhibition effect induced by up regulating miR-103a-3p alone, revealing that miR-103a-3p inhibits the malignant behavior of GSCs by declined FEZF1 expression.

CDC25A is an identified cell division cycle protein, which is required to enter S time [45], and the over-expression of this phosphatase accelerates the entrance to S time [46]. Our research showed that expression of CDC25A was remarkably increased in GSCs. Moreover, over-expression of CDC25A facilitated cell proliferation, migration and invasion, while inhibited apoptosis in GSCs. Consistent with our study, Wang XQ [47] reported expression of CDC25A elevated in hepatocellular carcinoma, which was significantly correlated with HCC tumor-node-metastasis staging and venous invasion. In addition, CDC25A was reported over-expressed and suppressed by miR-21 through a defined sequence in its 3′-UTR in colon cancer [48].

Moreover, we discovered that CDC25A was involved in a FEZF1-induced oncogenic effect in GSCs. Over-expression of FEZF1 could elevate CDC25A expression, while FEZF1 knockdown showed contrary effects. Luciferase assays and ChIP assays showed that FEZ1 increased promoter activity and bound to the promoter region of CDC25A, indicated that CDC25A was involved in FEZF1 regulation in GSCs.

Taken together, we revealed that the linc00152-miR-103a-3p-FEZF1-CDC25A axis manifested an important role in human glioma. Briefly, the miR-103a-3p over-expression induced by the knockdown of linc00152 could down-regulate the expression FEZF1, decreased FEZF1 hindered the promoter activities of CDC25A and inhibited malignant biological behavior in GSCs.

We further explored the molecular mechanisms of CDC25A oncogenic functions. Recent studies showed that CDC25A promoted PKM2-dependent β-catenin transactivation, which promotes the Warburg effect and tumorigenesis [49]. In addition, CDC25A was reported up-regulated in chondrosarcoma cells and played an important role in cell cycle progression and tumorigenesis of chondrosarcoma as an activator of CDK complexes [50]. Moreover, the activation of PI3K/AKT pathway participated in the glioma progression and various biological effects including proliferation, migration, invasion and apoptosis [51, 52]. The PI3K/AKT pathway inhibitors were discovered to exhibit efficacy against glioblastoma in clinically relevant mouse models [53]. In this work, we revealed that CDC25A over-expression activated the PI3K/AKT pathways in GSCs and knockdown of CDC25A manifested the opposite effects. Therefore, the reduced CDC25A induced by FEZF1 knocked down could attenuate the activity of PI3K/AKT pathways to inhibit the malignant behaviors of GCSs. The mechanism underlying tumor suppressive function of human glioma cells by linc00152 knockdown is schematically presented in Fig. 8e.

RETRACTED

## Conclusions

In summary, our research verified linc00152 facilitated cell proliferation, migration and invasion, while suppressed apoptosis in GSCs. MiR-103a-3p functioned as tumor suppressor by decreasing FEZF1 in GSCs. FEZF1 was downstream targets of miR-103a-3p, and CDC25A was a target of FEZF1. The significance of interaction among linc00152, miR-103a-3p, FEZF1 and CDC25A was highlighted for the first time. In addition, linc00152-miR-103a-3p-FEZF1-CDC25A axis might represent a promising therapeutic strategy for the treatment of human glioma.

## Methods

### Patients and glioma specimens

Grades of glioma were identified by neuropathologists according to WHO classification. Glioma specimens were divided into two groups: grade I–II glioma group (*n* = 10) and grade III–IV glioma group (*n* = 10). Normal brain tissues(NBTs) were used as the negative control group (*n* = 30). They were acquired from patients’ fresh autopsy material (donation from individuals who died in traffic accident and confirmed to be free of any prior pathologically detectable conditions).

### Cell culture

Human glioma cell lines (U87, U251) and human embryonic kidney (HEK) 293 T cells were purchased from the Chinese Academy of Medical Sciences (Beijing, China). U87 glioma cells and HEK-293 cells were cultured in Dulbecco’s modified Eagle medium (DMEM)/high glucose with 10% fetal bovine serum (FBS, Gibco, Carlsbad, CA, USA), U251 cells were cultured in DMEM/F12 medium with 10% FBS. All cells were maintained in a humidified incubator at 37 °C with 5% CO_2_.

### Isolation and identification of GSCs

GSCs were seperated as described previously [54, 55]. In a nutshell, GSCs were cultured in DMEM/F-12 medium (Life Technologies Corporation, Grand Island, NY, USA) appended to basic fibroblast growth factor (bFGF, 20 ng/mL, Life Technologies Corporation, Carlsbad, CA, USA), epidermal growth factor (EGF, 20 ng/mL, Life Technologies Corporation, Gaithersburg, MD, USA) and 2% B27 (Life Technologies Corporation, Grand Island, NY, USA). The serum-free medium was replaced every 2 days until the spheres were visible under microscopy. The spheres were centrifuged for 3 min at 1000 r.p.m. and harvested, then trypsinized into single-cell suspensions and plated into a 96-well plate for the limiting dilution assay and colon sphere formation by limiting dilution as described previously [56, 57]. For differentiation assay, sphere cells were plated onto glass coverslips coated with poly-L-ornithine (BD Biosciences, Franklin Lakes, NJ, USA) in medium containing 10% FBS for the differentiation assay. For immunostaining of undifferentiated spheres, cells were incubated with antibodies against Nestin and CD133 (1:100, Santa Cruz Biotechnology, Santa Cruz, CA, USA). For immunostaining of differentiated spheres, cells were stained with antibodies against GFAP (1:100, Abcam, Cambridge, MA, USA) and beta-tubulin III (1:100, Santa Cruz Biotechnology). The primary antibody complexes were visualized with anti-rabbit Alexa Fluor 488 and anti-mouse Alexa Fluor 555 secondary antibodies (Beyotime Institute of Biotechnology, Jiangsu, China). Nuclei were counterstained with 4′, 6-diamidino-2-phenylindole (DAPI).

RETRACTED

### Cell transfection and generation of stable transfected cells

Short-hairpin RNA directed against human linc00152 plasmid (sh-linc00152), short-hairpin RNA directed against human FEZF1 plasmid (FEZF1(−)), short-hairpin RNA directed against human CDC25A plasmid (CDC25A(−)) and their respective non-targeting sequence (negative control, NC) were synthesized (GenePharma, Shanghai, China). FEZF1 full length (FEZF1(+)) plasmid, CDC25A full length (CDC25A(+)) plasmid, and their respective non-targeting sequence (negative control, NC) were synthesized (GenScript, Piscataway, NJ, USA). Glioma cells were transfected in 24-well plates using Opti-MEM and Lipofectamine 3000 reagents (Invitrogen, CA, USA) according to the manufacturer’s instructions. Stable cell lines were selected applying Geneticin (G418; Invitrogen, CA, USA). Four weeks later, G418-resistant cell clones were established. The over-expression and the silence efficiencies were evaluated by quantitative real-time PCR (qRT-PCR). And then GSCs were isolated as previously described. To investigate the effect of linc00152 on GSCs, cells were divided into three groups: control group, sh-NC group (tansfected with empty plasmid) and sh-linc00152 group. To investigate the effect of FEZF1 on GSCs, cells were divided into five groups: control group, FEZF1(+)-NC group, FEZF1(+) group, FEZF1(−)-NC group and FEZF1(−) group. To investigate the effect of CDC25A on GSCs, cells were divided into five groups: control group, CDC25A(+)-NC group, CDC25A(+) group, CDC25A(−)-NC group and CDC25A(−) group.

RETRACTED

### Cell transfection of miRNAs

MiR-103a-3p agomir (pre-miR-103a-3p), miR-103a-3p antagomir (anti-miR-103a-3p) and their respective negative control molecules (pre-NC and anti-NC) were synthesized (GenePharma, Shanghai, China). To investigate the effect of miR-103a-3p on GSCs, cells were divided into five groups: control group, pre-NC group, pre-miR-103a-3p group, anti-NC group and anti-miR-103a-3p group. To investigate whether linc00152 mediated regulation of miR-103a-3p expression could regulate the behavior of GSCs, cells were divided into five groups: control group, sh-NC + pre-NC group (sh-NC stable transfected cells co-transfected with pre-NC), sh-linc00152 + pre-miR-103a-3p group (sh-linc00152 stable transfected cells co-transfected with pre-miR-103a-3p), sh-NC + anti-NC group (sh-NC stable transfected cells co-transfected with anti-NC) and sh-linc00152 + anti-miR-103a-3p group (sh-linc00152 stable transfected cells co-transfected with anti-miR-103a-3p). To investigate the mechanism of FEZF1 regulated by miR-103a-3p to effect the behavior of GSCs, cells were divided into five groups: control group, pre-NC + FEZF1-NC group (FEZF1-NC stable transfected cells co-transfected with pre-NC), pre-miR-103a-3p + FEZF1-NC group (FEZF1-NC stable transfected cells co-transfected with pre-miR-103a-3p), pre-NC + FEZF1 group (FEZF1 stable transfected cells co-transfected with pre-NC) and pre-miR-103a-3p + FEZF1 group (FEZF1 stable transfected cells co-transfected with miR-103a-3p).

### RNA and miRNA isolation and quantitative RT-PCR

Total RNA was isolated from the glioma tissues, NBTs and cells using Trizol reagent (Life Technologies Corporation, Carlsbad, CA, USA). The RNA concentration was determined by 260/280 nm absorbance using a Nanodrop Spectrophotometer (ND-100, Thermo, USA). One-Step SYBR PrimeScript RT-PCR Kit (Perfect Real Time) (Takara Bio, Inc., Japan) was used for qRT-PCR detection of linc00152 and mRNA of FEZF1 and CDC25A. cDNA from miRNAs was generated by using a TaqMan miRNA Reverse Transcription kit (Applied Biosystems, Foster City, CA, USA). qRT-PCR was carried out by using TaqMan Universal Master Mix II with Taq-Man microRNA assays of miR-103a-3p and U6 (Applied Biosystems, Foster City, CA, USA). U6 and GAPDH were employed as endogenous controls for miRNA and gene expression detection. Expressions were normalized to endogenous controls and relative quantification (2^−ΔΔCt^) method was used for fold changes’ calculating.

RETRACTED

### Cell proliferation assay

Cell proliferation was measured by conducting Cell Counting Kit-8 (CCK-8, Beyotime Institute of Biotechnology, Jiangsu, China) assay. After transfection efficacy was measured, GSCs were dissociated with Accutase (Life Technologies Corporation, Carlsbad, CA, USA), resuspended, and seeded in 96-well plates at 2000 cells per well. Cells per well were added 10 μl CCK-8 solution and cultured for 2 h at 37 °C. The absorbance was recorded at 450 nm on a SpectraMax M5 microplate reader (Molecular Devices, USA).

### Limiting dilution assay

Different amounts (2, 5, 10, 20, 50, 100, 200, 500) of GSCs were seeded into a 96-well plate. Serum-free conditional culture medium (25 μl) was added to each well every 2 days. The percentage of wells without neurospheres was enumerated. Then, a linear regression model was used to compare the slope of each group.

### Cell migration and invasion assay

Cells were resuspended in 200 μL serum-free medium at a density of 2 × 10^5^ cells/ml and placed in the upper chamber (or precoated with 80 μL of Matrigel solution (BD, Franklin Lakes, NJ, USA) for cell invasion assay) of the 24-well insert with 8 mm pore size. 600 μL of 10% FBS medium was added to the lower chamber. After incubation for 24 h, Cells had migrated or invaded to the lower side of the membrane were fixed and stained with 20% Giemsa. Stained cells were counted under a microscope in five randomly chosen fields and the average number was calculated.

### Apoptosis detection

Apoptosis was detected by Annexin V-APC/7-AAD (BD Biosciences). Cells were harvested added allophycocyanin (APC) and 7-aminoactinomycin D (AAD) following the instructions of the manufacturer. Cell samples were analyzed by flow cytometry (FACScan, BD Biosciences), and apoptotic fractions were recorded.

### Western blot analysis

Total proteins were isolated from cells with RIPA buffer on ice and were further analysed by SDS-PAGE and electrophoretically transferred to polyvinylidene difluoride membranes. After non-specific binding was prevented by 5% nonfat milk at room temperature for 2 h, membranes were embraced overnight at 4 °C by primary antibodies as below: FEZF1 (1:200, Santa Cruz Biotechnology),CDC25A(1:1000, Abcam, EUGENE, USA), PI3K, p-PI3K, AKT, p-AKT (1:1000, Cell Signaling Technology, Beverly, MA, USA) and GAPDH (1:1000, Santa Cruz Biotechnology). Then, incubated 2 h at room temperature with HRP-conjugated secondary antibodies. Immunoblots were visualized by ECL chemiluminescence detection system and the relative integrated density values were calculated by FLuor Chem2.0 software.

RETRACTED

### Dual-luciferase reporter assays

Potential miR-103a-3p binding sites of linc00152 and FEZF1 3′-UTR were predicted by bioinformatics tool Starbase (http://starbase.sysu.edu.cn/) and Target Scan (http://www.targetscan.org/). In brief, the fragment of linc00152 possessing the assumptive miR-103a-3p binding sites was cloned into a pmirGLO Dual-Luciferase Vector (Promega, Madison, WI, USA) to construct the reporter vector linc00152-wild-type (linc00152-Wt) (GenePharma, Shanghai, China). Analogously, the corresponding mutant of hypothetic miR-103a-3p binding sites was manufactured to form the reporter vector linc00152-mutated-types (linc00152-Mut) (GenePharma, Shanghai, China). The 3′-UTR fragment of FEZF1 gene and its mutant of the theoretical miR-103a-3p binding site were cloned into a pmirGLO Dual-Luciferase Vector to form the reporter vector FEZF1-3′-UTR-wild-type (FEZF1-3′-UTR-Wt) and FEZF1-3′-UTR-mutated-type (FEZF1-3′-UTR-Mut) (GenePharma, Shanghai,China), respectively. The pmirGLO vector(wild type fragments or mutated type fragments) and indicated miRNAs were transfected into HEK 293 T cells using Lipofectamine 3000. Relative luciferase activities were measured 48 h after transfection and firefly luciferase activity was normalized by renilla luciferase activity.

### Chromatin immunoprecipitation (Chip) assay

The Chip assay was carried out using the Simple Chip Enzymatic Chromatin IP kit (Cell Signaling Technology, Danvers, MA) following the manufacturer’s instructions. Cells were cross-linked with 1% formaldehyde for 10 min and then dealed with glycine for 5 min at room temperature. Cells were lysed with cold buffer containing PMSF and resuspended with cold PBS. Chromatin was digested by micrococcal nuclease and incubated for 20 min at 37 °C with frequent mixture. Lysates (2%) were employed as an input reference. Other immunoprecipitation samples were incubated overnight with normal rabbit IgG or anti-FEZF1 antibodies (Santa Cruz Biotechnology, CA, USA) at 4 °C with vibration. Protein G agarose beads were used to collect the chromatinimmune complex, and beads were scoured with low salt chip buffer and high salt chip buffer. DNA crosslinks were reversed by 5 mol/l NaCl and proteinase K at 65 °C for 2 h to purify. DNA was amplified by PCR applying the following DNA fragments: putative binding site 1 using the primers 5′-GGCTAAGAAGTGGTGGGAAAG-3′ and 5′-AGGGAGGGAATGCAATGAC-3′, generating a 211 bp product; putative binding site 2 using the primers 5′-GCTTTCTTCTTCCCCTCTCA-3′ and 5′-CCGACCTACACCTCTTACCC-3′, generating a 195 bp product; control using the primers 5′-TCTACCTCCTTCAGGGCTCA-3′ and 5′-TTTGGCCTTATCCTGTGGAC-3′, generating a 171 bp product.

RETRACTED

### Tumor xenografts in nude mice

In vivo study, the stable expressing cells were applied. Lentivirus encoding miR-103a-3p and its non-targeting sequence (negative control, NC) were generated using pLenti6.3/V5eDEST Gateway Vector Kit (Life Technologies Corporation, Carlsbad, CA, USA). The miR-103a-3p and short-hairpin RNA targeting human linc00152 were ligated into the pLenti6.3/V5eDEST vector and LV3-CMV-GFP-Puro vector (GenePharma, Shanghai, China), respectively. And then pLenti6.3/V5eDEST-miR-103a-3p and LV3-CMV-GFPPuro-sh-linc00152 vectors were generated. The ViraPower Packaging Mix was used to generate Lentivirus in 293FT cells. After infection, the stable expressing cells of miR-103a-3p (miR-103a-3p(+)), sh-linc00152 (linc00152(−)) were picked. The lentiviruses of miR-103a-3p(+) were transduced in linc00152(−) stably transfected cells to generate linc00152(−) + miR-103a-3p(+) cells.

The nude mice were divided into five groups: control group, linc00152(−)-NC + miR-103a-3p(+)-NC group, linc00152(−) group, miR-103a-3p(+) group and linc00152(−) + miR-103a-3p(+) group.

For subcutaneous implantation, every mouse was subcutaneously injected with 3 × 10^5^ cells in the right flank. Tumor volume was measured every 4 days using the formula: volume (mm^3^) = length × width2/2. The subcutaneous tumor-bearing mice were executed 40 days after injection. For survival analysis in orthotopic transplantation, 3 × 10^5^ cells were stereotactically transplanted into the right striatum of the mice. The number of survived nude mice was recorded every day and survival analysis was conducted applying KaplaneMeier survival curve.

### Statistical analysis

SPSS 18.0 statistical software was used for statistical analysis. All data are presented as the mean ± standard deviation (SD) from at least three independent replicates. Statistical analysis of data was performed using the Student’s t-test. Differences were considered to be statistically significant when *P* < 0.05.

## Additional file

Additional file 1: Figure S1. Isolation and identification of GSCs. **A**. a, c: Cells grew into spheres in serum-free medium. b, d: Spheres generated again from a single cell. **B**. Individual undifferentiated GSCs-87 and GSCs-251 stained for Nestin (green) and CD133 (red) by immunofluorescence analysis. **C**. Cell spheres were differentiated and then stained for GFAP (green) and β-tubulin III (red) by immunofluorescence analysis. Nuclei (blue) were labeled with DAPI. Images are representative of independent experiments (*n* = 5). Scale bars represent 20 μm. (TIFF 35029 kb)

## Abbreviations

3’UTR: 3’untranslated region
CCK-8: Cell counting kit-8
CDC25A: Cell division cycle 25A
ceRNA: Competing endogenous RNA
DMEM: Dulbecco’s modified Eagle Medium
FBS: Fetal bovin serum
FEZF1: Forebrain embryonic zinc finger protein 1
GSCs: Glioma stem cells
linc00152: Long intergenic non-coding RNA 152
mut: Mutation type
NBT: Normal brain tissue
qRT-PCR: Real-time quantitative polymerase chain reaction
wt: Wild type
